# Multi-channel feature fusion attention Dehazing network

**DOI:** 10.1371/journal.pone.0286711

**Published:** 2023-08-14

**Authors:** Changjun Zou, Hangbin Xu, Lintao Ye

**Affiliations:** East China Jiaotong University, Nanchang, China; University of Engineering & Technology, Taxila, PAKISTAN

## Abstract

Haze is a typical weather phenomena that has a significant negative impact on transportation safety, particularly in the port, highways, and airport runway areas. A multi-scale U-shaped dehazing network is proposed in this research, which is based on our multi-channel feature fusion attention structure. With the help of the feature fusion attention techniques, the model can focus on the intriguing locations with higher haze concentration area. In conjunction with UNet, it can achieve multi-scale feature reuse and residual learning, allowing it to fully utilize the feature information of each layer for image restoration. Experimental resulsts show that our technique performs well on a variety of test datasets. On highway data sets, the PSNR / SSIM / *L*_∞_ error performance over the novel technique is increased by 0.52% / 0.5% / 30.84%, 4.68% / 0.78% / 26.19% and 13.84% / 9.05% / 55.57% respectively, when compared to DehazeFormer, MIRNetv2, and FSDGN methods. The findings suggest that our proposed method performs better on image dehazing, especially in terms of *L*_∞_ error performance.

## Introduction

Haze is a common weather occurrence that limits visibility and poses a serious hazard to transportation safety. Haze affects many applications, including video surveillance and autonomous driving, and complex computer vision tasks such as image segmentation, visual detection, and visual identification. It can reduce the sharpness and contrast of images captured with image capture equipment, as well as cause color shift and a significant loss of image detail, making it difficult to acquire authentic image information.

Motivation: Heavy hazy weather is common throughout the spring and fall, which negatively affects both maritime and land transportation. Deep learning-based image dehazing is now feasible thanks to the quick development of deep learning-based image processing technologies. Investigating a deep learning-based image dehazing method is important from a practical standpoint. This technology will help to increase transportation safety, particularly for highway, rail, and watercraft safety.

Haze scattering causes a significant loss of image information collected by imaging sensors, severely limiting the value of image equipment applications. As a result, image dehazing is becoming more important with substantial research potential. Dehazing such images to increase image quality improves both transportation safety and the functionality of vision systems.

The dehazing algorithm is an image analysis and processing method that attempts to match the needs of a specific scenario, emphasize image details, and improve image quality. Image dehazing technology aims to lessen the impact of a hazy environment on image quality while also boosting image visibility, it is a difficult task in image processing and computer vision. Deep learning-based dehazing approaches have been an important study trend in the subject of dehazing in recent years, with the rapid expansion of artificial intelligence technology attracting the interest of many academics in the field of computer vision.

We discovered that the deep learning-based Feature Fusion Attention (FFA) technique works brilliantly in the area of image dehazing in earlier study [1]. The attention mechanism can greatly lower the system’s hardware requirements,especial for the mobile vehicles system [2, 3]. The basic goal of the deep learning attention mechanism, similar to the human selective visual attention mechanism, is to select the information that is more critical to the current task goal from a large amount of data. The attention method can help the model assign different weights to each component of the input and extract more critical information, allowing it to make more accurate decisions without increasing the model’s computation and storage overhead. Attention mechanisms are utilized in a variety of disciplines, including computer vision, image segmentation, image restoration, machine translation, speech recognition, image interpretation etc. The attention mechanism is simple and can make models more discriminating. As a result, the attention mechanism is well-suited to image dehazing tasks, especially when haze concentration distribution is uneven. According to our findings, the dehazing method based on the attention mechanism also has obvious benefits. Our contributions are as follows:

1. To achieve multi-scale intelligent image dehazing, an U-shaped Multi-channel Feature Fusion Attention Network (UMFFA) based on multi-channel feature fusion attention is proposed. Over the original Unet and FFA networks, our novel method improves PSNR/ SSIM/ *L*_∞_ error performance by 5.06%/ 3.40%/ 36.20%, 10.37%/ 6.46%/ 79.17%, respectively, on the Highway dataset.
2. An enhanced Multi-path Channel Pooling Attention (MCPA) structure is developed for the channel fusion module, which can recover more information than the original average pooling structure. The PSNR/ SSIM/ *L*_∞_ error performance improved by 0.19%/ 1.07% /2.70% respectively, after using multi-channel pooling on the Highways dataset.
3. A hybrid *L*_*H*_ loss function that takes into account the *L*_∞_ error is proposed, and the network’s *L*_∞_ error performance is greatly improved when compared to the original *L*_1_ loss function, effectively lowering the system’s *L*_∞_ error. When *β* = 0.002 is set, the PSNR/ SSIM/ *L*_∞_ error performance metrics improved by 2.07%, 1.48% and 16.37%, respectively, over the benchmark test.

Summary of our contributions: The idea of a multi-scale dehazing network based on multi-channel feature fusion attention is the main contribution of this paper. The approach of feature fusion attention is used to achieve efficient feature learning, and the multi-scale feature reuse as well as residual learning are realized by U-shaped structure in order to completely utilize the feature information of each layer for image restoration. Our multi-channel feature attention is used in feature learning to enable more efficient feature recovery. In order to solve the problem that the *L*_∞_ error cannot be effectively decreased in the current methodologies, a novel *L*_∞_ loss function is proposed. With obvious improvement, this function not only raises the PSNR/SSIM performance metrics but also greatly reduses the *L*_∞_ error.

Next, Sec. 2 will introduce the related research; Sec. 3 will introduce the new method proposed by us; Sec. 4 will introduce the test results, including ablation test and visual performance comparison; Sec. 5 will summarize this research.

## Related research

There are two sorts of image dehazing methods: conventional methods based on prior knowledge and intelligent dehazing methods based on deep learning.

Traditional dehazing methods, such as He’s Dark Channel Prior (DCP) method [4], Tan’s Maximum Contrast (MC) method [5], and Zhu’s Color Attenuation Prior (CAP) method [6] [7], Hue Disparity (HD) technique of Ancuti [8] and so on. The classic priori knowledge technique determines the priori connection between haze-free images and certain parameters in the atmospheric scattering model by doing feature analysis on a large number of haze-free images. However, such methods are not without flaws due to the limitation of the known priori information. For example, the dehazing performance isn’t ideal for hazy images with sky, and it can induce distortion in many cases.

As a result, deep learning-based intelligent dehazing algorithms are gaining more traction as a way to compensate for the lack of specific a priori drawbacks. The DehazeNet [9] model combines four priori dehazing algorithms: dark channel priori, maximum contrast dehazing, color attenuation, and chromaticity inconsistency-based dehazing. It uses a 4-layer convolutional neural network structure to estimate the atmospheric degradation model and improve the recovered image quality. While the AODNet [10] model allows end-to-end embedding into other models, such as lightweight Convolutional Neural Network(CNN). To increase the quality of texture information recovery and deliver better visually haze-free images. Cycle-Dehaze [11], does not rely on atmospheric scattering model parameter estimates. RefineDNet [12] divides the dehazing problem into two subtasks: visibility recovery and realism improvement, to combine the benefits of a priori-based and deep learning-based approaches. For example, before restoring vision, RefineDNet employs a dark channel in the first stage. The second step improves the first stage’s dehazing results by learning blurred and clear images in an adversarial fashion to improve realism.

DCPDN [13] is a multi-stage hierarchical deep learning network that employs a stage-based training technique in the training phase and a densely connected encoder-decoder network of edge pyramids for exact transmission mapping prediction. The EPDN [14] method, which is based on the global priority theory of visual perception and uses a pyramidal hierarchy to generate the adversarial network, does not use physical scattering models and instead uses a discriminator to direct the generator to create pseudo-realistic images at coarse scales, while the enhancer behind the generator is required to generate realistic dehazed images at fine scales. The image dehazing method based on the PCFAN [15] and the UNet architecture [16–18] effectively extracts the interdependent channel maps at different levels and can better recover image detail information. GridDehazeNet [19, 20] approach can alleviate the bottleneck problem commonly experienced in classic multi-scale methods and assist decrease artifacts in the final output. GCANet [21] uses smooth convolution instead of extended convolution to tackle the grid artifact problem. The haze-free images are directly recovered by the feature fusion attention network (FFA-Net) [22]. It is distinguished by its feature attention (FA) module [23], which integrates the channel and pixel attention methods, taking into account the fact that distinct channel features have entirely different weighting information and that haze is distributed unevenly over the image space.

Besides, there are still related technique, such as feature attention net for cell image segmentation [24], remote sensing image segmentation [25], image classification [26], style transfer [27], feature extraction [28], facial expression recognition [29], target feature captures [30], object detection [31] etc. In order to reduce the impact of hazy image and take into account the impact of depth in dehazing operation, the approaches based on physical models make use of the image depth information [32]. Images with various exposure levels are merged into haze-free images by adaptive structural decomposition based on multi exposure image fusion (MEF) scheme to each image block. Without the use of a physical model inversion of haze, the suggested image dehazing approach can successfully remove the visual damage brought on by haze [33]. The parameters of the linear scene depth model are trained with differentiable functions to produce the scene depth map of the remote sensing image, which is then used to estimate the atmospheric light of each fuzzy remote sensing image with the help of the associated scene depth map [34]. Using residual octave convolution, a network for dehazing remote sensing images is based on double self-attention (DOC) [35].

Existing techniques have the advantage of concentrating limited computational resources on the region of interest. However, it has been observed that the attention mechanism can yield good results in the case of uniform haze concentration distributions, such as FFA-Net [22]. The attention method, on the other hand, fails miserably in the case of agglomerate haze with rapidly shifting haze dispersion concentrations. In addition, we discovered in our research that the Unet-based multiscale learning method has some advantages in dealing with such situation, including the ability to successfully mix multiple scale feature information and a larger perceptual field. Furthermore, in channel attention, FFA-Net employs global averaging pooling, which smooths neighboring feature information. Multi-path channel pooling employs combination of global average and global maximum pooling, which improves network performance, according to our findings. As a result, we propose that multi-scale Unet be combined and improved with a multi-channel attention mechanism that effectively combines the benefits of both strategies.

## Our method

### UMFFA and the basic block

In neural networks, the attention mechanism is a resource allocation mechanism that prioritizes the allocation of computing resources to higher priority tasks while addressing the problem of information overload with limited computational resources. In general, the more parameters a model in a deep learning network contains, the more expressive the model is and the more information it holds. But this might lead to information overload. By introducing the attention mechanism, we may tackle the information overload problem by focusing on the vital information that is more critical to the current task and even filtering out the redundancy information, boosting the efficiency and accuracy of image enhancing processing.

Attention processes have been effectively applied in tasks such as image segmentation and super-resolution in the field of computer vision. Existing visual attention models are spatially based, with the feature maps of the final convolutional layer typically weighted. Instead, we present an approach based on multi-channel feature fusion attention called the U-shaped Multi-channel Feature Fusion Attention Network (UMFFA), whose structure is given in Fig 1. With the help of the multi-channel attention module and the pixel attention module, UMFFA can recover comprehensive multi-scale feature information. In comparison to the previous single-scale method, we observed that our new method can better cope with the uneven distribution of haze concentration in our tests.

**Fig 1:** Schematic diagram of UMFFA structure.

Because the perceptual fields of feature maps at different scales are different, more detailed information is recovered to the greatest extent possible during the fusing of information at multiple levels. Furthermore, the depth of the U-net can be adjusted freely, and a depth of four layers usually meets most requirements. UMFFA is made up of Residual Dense Attention Blocks (RDAB) that are connected in a U-shape. RDAB is made up of Basic Blocks connected by dense connection, with pixel-wise connections employed in the residual dense process, as seen in Fig 2. The gradient and residual information may be propagated more effectively, properly, and promptly when combined with the dense residual connection module, further improving network performance.

**Fig 2:** Composition of the RDAB and Basic Block.

The Basic Block is made up of a Residual Dense Block (RDB), Multi-path Channel Attention (MCA), and Pixel Attention (PA) blocks; the attention network adds residual connections after MCA and PA to speed up the propagation of residual and gradient information, as seen in Figs 2 and 3. Local residual learning and feature attention modules are part of a basic block structure. Local residual learning modules enable it to skip through less essential data, such as less cloudy or low-frequency regions. The backbone network architecture can focus on more effective critical information thanks to the various local residual connections.

**Fig 3:** Multi-path channel attention and pixel attention modules.

MCA: In the previous channel connection attention module [22], average pooling was used to calculate channel weight. However, average pooling tends to smooth edges and lose detail information. As a result, we added another maximum pooling path to the improved Multi-path Channel Attention module in order to maintain more precise information. The convolution and activation layers are applied after the average and maximum pooling layers have been combined. This strategy enables more efficient detail acquisition and, as a result, increased learning efficiency.

PA: The pixel attention module uses a convolution and activation layer in sequence, as well as pixel-wise weighting and residual multiplication. The network treats distinct features and pixels unequally in the attention module, allowing for more flexibility in processing diverse types of data and extending the representation potential of convolutional neural networks. The feature weights in the Features Fusion Attention(FFA) layer of multiple levels of features structure are adaptively learned from the Feature Attention (FA) module, which gives essential features higher weights. This structure can also store and pass on shallow data to deeper layers.

### Multi-path Channel Attention module

The Multi-path Channel Attention (MCA) module primarily determines the weights of each channel based on the input feature information. Not only global average weights, but also global maximum pooling weights are produced in this module. This method allows for the collection of more specific information. The input and output images in the attention module have dimensions of *C* × *H* × *W* and *C* × 1 × 1, respectively. After applying global average and maximum pooling to the input data, we can obtain:

$$\begin{array}{c} g_{a}=H_{ap}\left(F_{c}\right)=\frac{1}{H\times W}\sum_{i=1}^{H}\sum_{j=1}^{W}X_{c}\left(i,j\right) \end{array}$$ (1)

$$\begin{array}{c} g_{m}=H_{mp}\left(F_{c}\right)=Max\left[X_{c}\left(i,j\right)\right] \end{array}$$ (2)

Where *H*_*ap*_, *H*_*mp*_ are Global Average Pooling and Global Max pooling functions respectively; *F*_*c*_ is the input; *X*_*c*_ is the input image; *H*,*W* are the height and width dimensions of the input image respectively.

Pooling layer has the function of reducing information redundancy and noise. Enhance the model’s rotational and scale invariance, decrease the amount of computation required, and prevent over-fitting. Maximize pooling could retain the main features, highlight the foreground (the depth of the general foreground is deeper than the background), and extract the texture information of the features. Average pooling could preserve background information and highlight background information.

Then, it goes to the convolution layer and activation layer after pooling and point-wise splicing, we get:

$$\begin{array}{c} CA_{c}=\sigma \left[Conv\left[\delta \left[Conv\left(Concat\left(g_{a},g_{m}\right)\right)\right]\right]\right] \end{array}$$ (3)

where *σ* and *δ* are the Relu and Sigmoid activation functions, respectively; Concat is the pixel-wise splicing; and Conv is the 1×1 convolution. Finally, the weights and the inputs are multiplied pixel-wise to obtain the final channel-aware output.

$$\begin{array}{c} F_{c}^{*}=F_{c}⊗CA_{c} \end{array}$$ (4)

where ⊗ is the point-wise multiplication, the detailed structure is shown in Fig 3. According to our method, the input image enters the global average pool and global maximum pool, respectively, before moving on to the convolution layer and activation layer for MCA. The output of MCA is produced by multiplying the weight gained by the input and output images. The input of PA is the output of MCA. After activation and 1x1 convolution, the acquired weight is multiplied by the input to produce the PA output.

### Pixel attention module

The Pixel Attention module concentrates on the pixel weight, or the haze concentration distribution at each pixel. The pixel attention module detects haze distribution over the entire image space and uses this information to execute targeted dehazing calculations. The input-output image shape of the pixel attention module changes from *C* × *H* × *W* to 3 × *H* × *W*. This output also contains the RGB per color component weights; when utilizing the MCA output as the PA input, we get:

$$\begin{array}{c} PA=\sigma [Conv\left[\delta \left[Conv\left(F_{c}^{*}\right)\right]\right]] \end{array}$$ (5)

Where $F_{c}^{*}$ is the output of the MCA; *σ* and *δ* are the Relu and Sigmoid activation functions, respectively; and Conv is the 1 × 1 convolution. Finally, the output of the final pixel-aware module is obtained after multiplying the weights with the input pixel by pixel as follows.

$$\begin{array}{c} F=F^{*}⊗PA \end{array}$$ (6)

Multi-path Channel Attention Weight and Pixel Attention Weight example are shown in Figs 4 and 5.

**Fig 4:** Input and pixel channel attention weight. (a) Input and (b) Pixel channel weight.

**Fig 5:** Multi-path channel attention weight.

### Hybrid loss function

UMFFA network adopts a hybrid loss function composed of *L*_1_ error and *L*_∞_ error, which improves the instability of *L*_∞_ error compared with the original Unet and FFA network. Meanwhile the PSNR / SSIM performance of our UMFFA is improved slightly, but the *L*_∞_ error has decreased significantly, indicating the evident benefits of the enhanced network.

(1) *L*_1_-Norm

*L*_1_- Norm is one of the most common norms, which is defined as follows:

$$\begin{array}{c} ∥x∥=\sum_{i=1}\left|x_{i}\right| \end{array}$$ (7)

The *L*_1_-norm can be used to measure the difference between two vectors, such as the Mean Absolute Error (MAE):

$$\begin{array}{c} MAE\left(x_{1},x_{2}\right)=\frac{\sum_{i=1}^{n}\left|x_{1i}-x_{2i}\right|}{n} \end{array}$$ (8)

(2) *L*_∞_-Norm

*L*_∞_-Norm is mainly used to measure the maximum value of vectors. It is defined as:

$$\begin{array}{c} {∥x∥}_{\infty }=\sqrt{\sum_{i}x{}_{i}^{\infty }},\left(x=x_{1},x_{2},...,x_{n}\right) \end{array}$$ (9)

In general, it can be expressed by the following formula:

$$\begin{array}{c} {∥x∥}_{\infty }=max(|x_{i}\left|\right) \end{array}$$ (10)

A very good feature of *L*_∞_-norm is that it is independent of the dimension of the vectors. This feature has certain advantages in comparing error vectors of different dimensions.

(3) *L*_*H*_ Hybrid loss function

The *L*_*H*_ Hybrid loss function is defined as:

$$\begin{array}{c} \left\{ \begin{array}{cc} L_{H} & =\alpha \cdot L_{1}+\beta \cdot L_{\infty }\\ \alpha +\beta & =1 \end{array}\right. \end{array}$$ (11)

In practice, we usually use mean absolute error instead of summation of absolute error in order to avoid the correlation between *L*_1_-norm and vector dimension. However, the direct use of *L*_1_-norm may reduce the average error, while the absolute error of some pixels may be still huge. This situation does occur. Because the *L*_1_-norm only reduces the average error, there is no limit to the error of a single pixel. Therefore, we need a new loss function that can not only reflect the overall error, but also effectively reduce the maximum error of a single pixel, so as to further improve the quality of image recovery.

The *L*_∞_-norm just satisfies this requirement, which allows us to easily compare the max error between a single pixels, which is independent of the number of vector dimension. Therefore, we proposed a hybrid error loss function combining *L*_1_-norm and *L*_∞_-norm, which can not only ensure the overall error of the image, but also effectively reduce the maximum error between individual pixels. Through our tests and analysis, it is found that the recommended value range of *β* is [0.002, 0.1]. Too large or too small will deteriorate the performance of the network.

### Implementation details

The feature attention module and our proposed UMFFA takes into account the possible uneven distribution of haze concentration on images, it could achieve weighted fusion of different channels and pixels through the attention mechanism. It also makes use of Unet’s multi-scale learning framework to build a number of perceptual fields capable of realizing different levels of feature information and residual information propagation.

The backbone network in UMFFA is shaped like Unet, and its depth may be adjusted freely. We observed that using 64 input feature maps and four levels of depth can offer good results after comparison tests. The number of feature maps doubles with each depth layer. Average pooling is employed in the downsampling procedure, and nearest neighbor interpolation is used in the upsampling.

In Unet’s basic block, RDAB consists of MCA and PA attention modules, and it maintains the basic residual dense connection structure with the depth of the dense residual connection set to 3 layers.

In MCA and PA, we employ convolutional layers to minimize feature map number, and the feature map number reduction ratio is 8. The convolutional kernel size for MCA and PA is 1 × 1, 3 × 3, respectively. The pooling functions in multichannel attention are average pooling and maximal pooling, respectively. The activation functions are Relu and Sigmoid, respectively.

In MCA output, the final output channel number is 1. But in PA output, it is 3, which represents the RGB component weights of the different color channels. During the training process, the preprocessor evenly crops the input images to size 128 × 128 for distinct training sets, with no overlap between images. The training output is the same size as the original input image.

## Experiment results

### Training platform, data, and performance evaluation metrics

This research compares the standard datasets in order to validate this dehazing strategy. I-Haze [36], O-Haze [37], NH-Haze [38] and Reside-Out [39] are the test datasets. We also proposed the Highway dataset to further validate the performance of different approaches in the scenario of uneven haze concentration distribution. The non-uniform haze concentration distribution is generated by a fog equation combined with a stochastic method in this dataset, which primarily uses the highway image as the background. It has 1200 sets of training images and 100 sets of test images, and some of the example images are displayed in Fig 6.

**Fig 6:** Highway dataset. (a) Ground truth and (b) Hazy image.

The main training performance evaluation metrics are PSNR, SSIM, and *L*_∞_ error. PSNR is a peak signal-to-noise ratio that serves as an objective measure for image evaluation. PSNR is the most popular and widely used approach for evaluating image quality objectively. The structural similarity index (SSIM) is a complete image quality evaluation metrics that compares image brightness, contrast, and structure. The training platform and related parameters employed in this technique are shown in Table 1.

**Table 1:** Training platform and related parameters.

CPU	Intel i9 12900K
GPU	RTX3080
CPU Memory	64G, DDR5, 4800MHZ
GPU Memory	GDDR6 12G
Operation System	Windows 10
Training platform	Keras 2.7

Training settings and outcomes: Optimizer is Adam, learning rate = 0.001, *β*_1_ = 0.9, *β*_2_ = 0.999, and Keras version 2.7 training platform. In the experiments comparing the performance of other methods, the comparison methods were replicated according to the literature, and the training process was conducted on the same platform and same data set. The number of iterations in the training procedure is 1000, and the epoch is 500.

### Comparison with existing methods

Comparison with existing methods: Our proposed UMFFA approach delivers good results on numerous diverse datasets, as shown in Table 2. The best outcome is denoted by the bold font, while the second-best result is denoted by the Italic font. Our method has shown better outcomes on many data sets when compared to numerous other exixting methods. With the exception of a modest decline in performance on certain data sets. Specifically, all of the metrics are optimal on the I-Haze, Highway, and Reside-Out datasets; on the NH-Haze dataset, only the *L*_∞_ error ranks second, and the rest of the metrics are also optimal; on the O-Haze dataset, the performance is not that satisfacotry, with the PSNR metric ranking third, the *L*_∞_ error ranking second, and the SSIM metric ranking first.

**Table 2:** Comparison of the performance of different methods.

Method	Metrics	I-Haze	O-Haze	NH-Haze	Highway	Reside-out
Dehaze	PSNR	17.1536	18.4663	14.2850	18.8508	21.3887
	SSIM	0.7551	0.5990	0.3876	0.5184	0.7776
	*L*∞ error	0.4710	0.4652	0.6505	0.7106	0.4872
AOD	PSNR	18.1055	20.0963	14.9713	19.5627	23.3680
	SSIM	**0.7998**	0.6836	0.5337	0.7079	0.9132
	*L*∞ error	0.3980	0.4501	0.5496	0.6544	0.2628
Unet	PSNR	17.0351	19.0942	14.0307	24.1866	24.2640
	SSIM	0.7377	0.6203	0.4721	0.8224	0.9021
	*L*∞ error	0.4390	0.4159	0.6608	0.4511	0.2642
FFA	PSNR	18.0209	*19.8969*	14.0055	22.8338	24.2237
	SSIM	0.7951	0.6699	0.5196	0.7963	0.9100
	*L*∞ error	0.4318	**0.3693**	0.6666	0.5934	0.2916
ClarifyNet	PSNR	19.5482	19.6951	15.7397	25.4749	25.2920
	SSIM	0.7410	0.6831	*0.5770*	0.7903	0.9115
	*L*∞ error	0.2279	0.3280	0.4943	0.5246	0.2004
FSDGN	PSNR	18.0664	*20.8363*	15.6362	24.6001	25.1109
	SSIM	0.7617	**0.7135**	0.5467	0.8299	0.9189
	*L*∞ error	0.1759	**0.2375**	0.4116	0.4717	0.1053
MIRNetv2	PSNR	*18.1267*	19.8433	15.5549	27.2154	*25.6469*
	SSIM	0.7763	0.6909	0.5442	0.9054	**0.9340**
	*L*∞ error	**0.1375**	0.2460	*0.3218*	*0.3826*	**0.0896**
DehazeFormer	PSNR	**18.9486**	**20.9181**	*16.1253*	*28.4036*	25.0250
	SSIM	0.7535	0.7070	0.5700	*0.9079*	0.9095
	*L*∞ error	0.1457	0.2439	**0.3134**	0.3967	0.0944
Our method	PSNR	17.6893	20.5230	**16.3832**	**28.5510**	**25.6885**
	SSIM	0.7638	*0.7109*	**0.5837**	**0.9125**	*0.9297*
	*L*∞ error	*0.1399*	*0.2397*	0.3416	**0.3032**	*0.0908*

From this results, it can be stated that, while the new technique does not produce the best results in all datasets, it does so in the majority of them, and its performance is significantly enhanced when compared to the original FFA and Unet methods as well as many of the recent advanced methods, demonstrating the new method’s benefits.

### Ablation tests

A series of ablation tests was devised to verify the influence of different structures in this method on the final performance. The ablation tests were separated into four groups based on different settings, as indicated in Table 3, with the UMFFA technique serving as the baseline and the Unet, FFA, and RDN methods serving as comparison tests.

**Table 3:** Ablation test setup.

Method	Unet module	FFA module	RDB module
UMFFA	✓	✓	✓
Unet	✓	X	X
FFA	X	✓	X
RDN	X	X	✓

The metrics of several procedures in the ablation test are quantitatively compared in Table 4 and Fig 7. On the Highway data set, UMFFA is the benchmark group, with PSNR/ SSIM/ *L*_∞_ errors of 25.4749/ 0.8513/ 0.3312, respectively, where the greater the first two metrics, the better the performance, and the smaller the last metrics, the better the performacne. The PSNR/ SSIM/ *L*_∞_ error of the Unet is 24.1866/ 0.8224/ 0.4511, compared to the UMFFA approach, where the PSNR/ SSIM reduces by 5.06%/ 3.40%, and the *L*_∞_ error increased by 36.20% respectively.

**Fig 7:** Changes in performance metrics of different methods in ablation tests. (a) PSNR and (b) SSIM.

**Table 4:** Comparison of ablation test performance metrics on the Highway data set (average on last 20 results).

Method	PSNR	SSIM	*L*_∞_ loss
UMFFA	25.4749	0.8513	0.3312
Margin	-	-	-
Unet	24.1866	0.8224	0.4511
Margin	-5.06%	-3.40%	36.20%
FFA	22.8338	0.7963	0.5934
Margin	-10.37%	-6.46%	79.17%
RDN	20.7830	0.7604	0.5740
Margin	-18.42%	-10.68%	73.31%

The FFA method’s PSNR/ SSIM/ *L*_∞_ error is 22.8338/ 0.7963/ 0.5934, with the PSNR/ SSIM lowered by 10.37%/ 6.46% and the *L*_∞_ error increased by 79.17%. Similarly, the PSNR/ SSIM/ *L*_∞_ error was 20.7830/ 0.7604/ 0.5740 for the RDN method compared with the UMFFA method, in which the PSNR/ SSIM decreased by 18.42%/ 10.68% and the *L*_∞_ error increased by 73.31% respectively.

The performance of Unet is the closest to the UMFFA results in these three sets of ablation comparison experiments, demonstrating that this multi-scale residual learning structure has a favorable influence on boosting the dehazing performance. Although the FFA method’s outcomes are second to the Unet method’s, the FFA method’s *L*_∞_ error is the biggest of the four techniques, demonstrating that the FFA method does not properly control the *L*_∞_ error on its own.

### Influence of *β* in the loss function on the performance metrics

Five sets of tests were set up for comparison in order to further verify the influence of *β* in the loss function on the PSNR/ SSIM/ *L*_∞_ performance metrics and to establish the optimal range of in these five sets of trials. *β* was changed between [0, 0.3], while the baseline group was set as *β* = 0. The result in Table 5, Figs 8 and 9 show that as *β* grows, all performance metrics improves. For example, when *β* is in the range of [0.002, 0.1].

**Fig 8:** Effect of different *β* on the performance metrics PSNR/SSIM. (a) PSNR and (b) SSIM.

**Fig 9:** The effect of *β* on the performance metrics *L*∞ error.

**Table 5:** Influence of *β* on performance metrics.

Method	PSNR	SSIM	*L*_∞_ loss
UMFFA *β* = 0	24.9591	0.8389	0.3960
Margin	-	-	-
UMFFA *β* = 0.002	25.4749	0.8513	0.3312
Margin	2.07%	1.48%	-16.37%
UMFFA *β* = 0.01	25.4088	0.8461	0.3301
Margin	1.80%	0.86%	-16.63%
UMFFA *β* = 0.1	25.1041	0.8438	0.3033
Margin	0.58%	0.59%	-23.40%
UMFFA *β* = 0.3	24.1297	0.7828	0.3840
Margin	-3.32%	-6.68%	-3.02%

As we can see, when *β* = 0.002, the PSNR/ SSIM/ *L*∞ performance metrics rises to 25.4749/ 0.8513/ 0.3312, compared to 24.9591/ 0.8389/ 0.3960 in the benchmark test, and performance improves by 2.07%/ 1.48%/ 16.37%, respectively. As *β* continues to rise, such as *β* = 0.1, the PSNR/ SSIM/*L*_∞_ performance metrics is 25.1041/ 0.8438/ 0.3033; while the *L*_∞_ performance metrics has increased, the PSNR/ SSIM metrics performance has dropped; While *β* = 0.3, the PSNR/ SSIM clearly deteriorates. As a result, we suggest that the acceptable range of *β* is [0.002, 0.1], with too small *β* it will has insignificant influence on the results, too large will leads to deterioration of other performance metrics.

### Multi-path channel pooling

Because global average pooling is employed in the channel attention in prior FFA approaches, this processing can cause edge smoothing and result in the loss of details information. As a result, our new method includes a maximum average pooling path in the channel attention module to improve detail loss, which combines average and maximum pooling. The performance metrics are enhanced with our multi-path channel pooling. The influence of applying multi-path pooling and average pooling on the Highway and I-Haze datasets, respectively, are shown in Tables 6 and 7.

**Table 6:** Comparison on Highway dataset with multi-channel pooling.

Method	PSNR	SSIM	*L*_∞_ loss
UMFFA with Multi-Channel Pooling	25.4749	0.8513	0.3312
Margin	-	-	-
UMFFA with Single Channel Pooling	25.4271	0.8422	0.3401
Margin	-0.19%	-1.07%	2.70%

**Table 7:** Comparison results with multi-channel pooling on the I-Haze dataset.

Method	PSNR	SSIM	*L*_∞_ loss
UMFFA with Multi-Channel Pooling	19.5482	0.8080	0.2914
Margin	-	-	-
UMFFA with Single Channel Pooling	19.3552	0.8080	0.3401
Margin	-0.99%	0.00%	3.24%

The PSNR/ SSIM/*L*_∞_ performance metrics on the Highway dataset are 25.4749/ 0.8513/ 0.3312, respectively, while the performance metrics without multi-path channel pooling are 25.4271/ 0.8422/ 0.3401, and the performance metrics with multi-path channel pooling are improved by 0.19%/ 1.07%/ 2.70%, respectively. The I-Haze dataset showed similar results, with performance metrics improved by 0.99% /0.00%/ 3.24% after using multi-path pooling, indicating that multi-path pooling can help boost model performance to certain level.

### Visual performance comparison

This experiment compares the visual performances of various methods on the datasets I-Haze and Highway. I-Haze is a real indoor dehazing test dataset with a relatively uniform haze concentration distribution, whereas Highway is a dehazing test dataset generated by haze scattering formation theory. This datasets is primarily comprised of highway sceneries with a non-uniform haze concentration distribution. These two datasets can be used to verify the dehazing algorithm’s performance.

Figs 10–13 show the results of the ClarifyNet [40], FSDGN [41], MIRNetv2 [42], DehazeFormer [43], and UMFFA techniques on these two datasets, respectively. In all of the cases, the UMFFA technique produces the best outcomes. The performance of the methods for the I-Haze dataset is often worse than that of the Highway dataset. The performance metrics of the tested dehazing algorithms improved when compared to the inputs, as shown in Figs 10 and 11, however the improvement is not considerable. And, as shown in Figs 12 and 13, our methods are generally superior than the others, particularly our proposed UMFFA method, which achieves the best results. The PSNR/ SSIM/ *L*_∞_ metrics are enhanced greatly, respectively, in these two sets of findings, indicating that the performance metrics effect is quite considerable. And it can be seen from these two sets of visual comparisons that after dehazing with UMFFA, the images grow sharper, and the result is very close to the Groud Truth image, with the dehazing result being extremely evident.

**Fig 10:** Image 109 from dataset I-Haze.

**Fig 11:** Image 132 from dataset I-Haze.

**Fig 12:** Image 21 from dataset Highway.

**Fig 13:** Image 28 from dataset Highway.

## Conclusion

In this paper, we proposed a U-shaped multi-channel feature fusion attention network that combines Unet with multiscale architecture and feature fusion attention mechanism to accomplish non-uniform distribution image dehazing. The attention network adds residual connections after MCA and PA to speed up the propagation of residual and gradient information. Local residual learning and feature attention modules are part of a basic block structure. Local residual learning modules enable it to skip through less essential data, such as less cloudy or low-frequency regions. The backbone network architecture can focus on more effective critical information thanks to the various local residual connections. We also proposed a non-uniform haze concentration distribution dataset based on highway scenes to test the perfromance of the new technique on non-uniformly distributed haze datasets. On the testing datasets, the new method outperforms on PSNR/ SSIM/*L*_∞_ error metrics, respectively, with a significant improvement in performance, especially for *L*_∞_ error. This method is more effective for non-uniform distribution image dehazing than many other methods.

In order to solve the problem that the *L*_∞_ error cannot be effectively decreased in the current methodologies, a novel *L*_∞_ loss function is proposed concurrently. With obvious improvements, this new loss function not only raises the PSNR/SSIM performance metrics but also greatly reduses the *L*_∞_ error. In the meanwhile, we present a multi-path channel attention structure that combines average pooling and maximum pooling path. The PSNR/ SSIM/ *L*_∞_ error performance metrics on the Highway and I-Haze datasets are significantly improved, when compared to the original average pooling attention structure, demonstrating the superiority of our new method.

## Supporting information

S1 File (RAR)
